# Exosomes Derived From MicroRNA-148b-3p-Overexpressing Human Umbilical Cord Mesenchymal Stem Cells Restrain Breast Cancer Progression

**DOI:** 10.3389/fonc.2019.01076

**Published:** 2019-10-22

**Authors:** Lei Yuan, Yuqiong Liu, Yunhui Qu, Lan Liu, Huixiang Li

**Affiliations:** ^1^Department of Pathology, The First Affiliated Hospital of Zhengzhou University, Zhengzhou, China; ^2^School of Basic Medical Sciences, Zhengzhou University, Zhengzhou, China

**Keywords:** miR-148b-3p, TRIM59, breast cancer, human umbilical cord mesenchymal stem cell, exosomes

## Abstract

Exosomes derived from human umbilical cord mesenchymal stem cells (HUCMSCs) expressing microRNAs (miRs) have been highlighted as important carriers for gene or drug therapy. Hence, this study aimed to explore the role of exosomal miR-148b-3p from HUCMSCs in breast cancer. Clinical samples subjected to RT-qPCR detection revealed that miR-148b-3p was poorly expressed, while tripartite motif 59 (TRIM59) was highly expressed in breast cancer tissues. Online analyses available at miRanda, TargetScan, and miRbase databases revealed that miR-148b-3p could bind to TRIM59, while dual-luciferase reporter gene assay further verified that TRIM59 was a target gene of miR-148b-3p. Next, miR-148b-3p mimic or inhibitor and siRNA against TRIM59 were delivered into the breast cancer cells (MDA-MB-231) to alter the expression of miR-148b-3p and TRIM59 so as to evaluate their respective effects on breast cancer cellular processes. Evidence was obtained demonstrating that miR-148b-3p inhibited cell proliferation, invasion, and migration, but promoted cell apoptosis in breast cancer by down-regulating TRIM59. Next, MDA-MB-231 cells were co-cultured with the exosomes derived from HUCMSCs expressing miR-148b-3p. The results of co-culture experiments demonstrated that HUCMSCs-derived exosomes carrying miR-148b-3p exerted inhibitory effects on MDA-MB-231 progression *in vitro*. *In vivo* experimentation further confirmed the anti-tumor effects of HUCMSCs-derived exosomes carrying miR-148b-3p. Taken together, HUCMSC-derived exosomes carrying miR-148b-3p might suppress breast cancer progression, which highlights the potential of exosomes containing miR-148b-3p as a promising therapeutic approach for breast cancer treatment.

## Introduction

Breast cancer is a common malignant tumor and the leading cause of cancer-related death in females. Unfortunately, the death toll surpassed 600,000 deaths and ~2 million new cases were diagnosed in 2018 worldwide (1). Breast cancer is characterized by its prominent heterogeneity on molecular phenotypes, clinical features, and tissue pathology, all of which reflect as higher morbidity, as well as an increased tendency to acquire breast cancer at younger ages in recent years (2, 3). Mesenchymal stem cells (MSCs), adult multipotent cells that possess the ability to differentiate and self-renew, are associated with the tumor microenvironment and tumor progression, and have been previously highlighted to serve as potential cytokines for future tumor therapy (4).

Human umbilical cord MSCs (HUCMSCs) are non-hematopoietic progenitor cells with multipotency capable of differentiating into different cell lineages, which could suppress the apoptosis of stromal cells through secretion of growth factors (5). A previous study has highlighted the inhibitory role of HUCMSCs in tumor formation of breast cancer by direct communication and internalization between cells (6). Meanwhile, exosomes from HUCMSCs (HUCMSCs-exo) have also been shown to actively participate in facilitating endothelial cell migration, proliferation, and tube formation (7).

Exosomes are recognized as secreted micro-vesicles carrying proteins, mRNAs, and miRs by bodily fluids, which stimulate immune responses, and accelerate communication among cells (8, 9). Additionally, exosomal microRNAs (miRs) secreted by cancer cells have been implicated in the regulation of tumor metastasis and development. For example, miR-105 has been previously reported to serve as an effective promoter of migration in breast cancer (10). MiRs are a form of endogenous and short non-coding RNA molecule with the length of around 18–25 nucleotides, which play regulatory roles in several genes and multiple pathways associated with pathological and physiological processes (11). Moreover, a recent study highlighted the involvement of miRs in the tumorigenesis and tumor invasiveness of breast cancer (12). As an important member of the miR-148/152 family, miR-148b-3p has been reported to exert a tumor suppressive role in glioma (13). Meanwhile, miR-148b-3p has also been identified to serve as a suppressor of metastasis in gastric cancer through suppression of the Dock6/Rac1/Cdc42 axis (14). Moreover, TRIM59, which forms part of the tripartite motif (TRIM) family, has been implicated in the regulation of the development of human diseases, such as cancers (15). In addition, elevation of TRIM59 has been detected in numerous malignant tumors, including breast cancer (16).

Based on the literature and findings, we proposed the hypothesis that HUCMSC-derived exosomes may transfer miR-148b-3p to breast cancer cells. As TRIM59 was predicted to be the target of miR-148b-3p by online prediction analyses, we speculated that miR-148b-3p could mediate the progression of breast cancer by targeting TRIM59 gene. Hence, the current study aims to validate if the aforementioned hypothesis was valid and to further explore the mechanisms by which exosomal miR-148b-3p suppresses the development of breast cancer through regulation of TRIM59 expression.

## Materials and Methods

### Study Subjects

A total of 40 breast cancer tissues and adjacent normal tissues were collected from breast cancer patients (age range 39–61 years; mean age 50.55 ± 6.01 years) who had previously undergone operative procedures at the First Affiliated Hospital of Zhengzhou University. All specimens were pathologically confirmed as primary breast cancer. All enrolled patients were yet to receive any radiotherapy or chemotherapy prior to their operation. All collected specimens were preserved at −80°C in a refrigerator.

### Cell Culture

Normal mammary epithelial cell line MCF-10A and breast cancer cell lines MDA-MB-231, MDA-MB-468, MCF-7, and MDA-MB-453 (Shanghai Life Science Institute of Chinese Academy of Sciences, Shanghai, China) were cultured with Dulbecco's modified eagle medium (DMEM) or Roswell Park Memorial Institute (RPMI)-1640 containing 10% fetal bovine serum (FBS) (Gibco, Grand Island, NY, USA) in 5% CO_2_ at 37°C. The complete medium was changed every 2–3 days. When cell confluence had reached 80%, the cells were detached with routine trypsin and passaged. Cells in the logarithmic phase of growth were used for subsequent experimentation.

### Cell Treatment

Breast cancer cells or HUCMSCs were transfected in accordance with the instructions of the Lipofectamine 2000 Transfection Reagent (11668-019; Invitrogen, Carlsbad, CA, USA) with miR-148b-3p mimic (4464066), miR-148b-3p inhibitor (4464084), TRIM59 overexpression plasmid (pcDNA3.1-TRIM59), siRNA targeting TRIM59 (siRNA-TRIM59; AM16708) or their negative controls including NC-mimic (4464060), NC-inhibitor (4464076), TRIM59-NC (pcDNA3.1-NC), and siRNA-NC (4390843). All the above-mentioned sequences and plasmids for transfection were purchased from Thermo Fisher Scientific (Waltham, MA, USA).

More specifically, the cells at the logarithmic phase of growth were trypsinized and triturated into a single cell suspension, seeded into a 6-well, and transfected once the cells had reached ~80% confluence. The cells were cultured at 37°C with 5% CO_2_ and saturated humidity after transfection. After 48 h, the medium was renewed with RPMI-1640 complete medium for further 24–48 h culture for follow-up experiments.

### HUCMSC Isolation and Identification

HUCMSCs were isolated from the fresh human umbilical cords which were obtained after full-term pregnancy cesarean section. A primary culture of HUCMSCs was conducted based on the standard procedure. Initially, the umbilical cords were washed with 75% ethanol and then cultured with DMEM containing 1% L-glutamine, 10% FBS, and 100 μg/mL streptomycin and penicillin. Next, the umbilical cords were sliced into small pieces (3–5 mm) and cultured at 37°C and with 5% CO_2_. The cells were subsequently detached with trypsin and sub-cultured when cell confluence reached 80–90%. Light microscopy was employed to analyze the cellular morphology.

Flow cytometry was performed to analyze the immunophenotypic features of HUCMSC. Initially, the cells were detached by trypsin for 2–4 min, blocked with 10% normal goat serum, and then cultured with a series of fluorescein isothiocyanate (FITC) dyes-labeled human monoclonal primary antibodies CD14, CD19, CD29, CD34, CD44, CD45, CD73, CD90, HLA-A, B, C, and HLA-DR (dilution ratio of 1:100; BioLegend, San Diego, CA, USA) for 30 min. Then, the cells were resuspended in 10% normal goat serum. At last, a CyAn ADP Analyzer (Beckman Coulter, Brea, CA, USA) was utilized for cell analyses.

### HUCMSC Exosome (HUCMSC-exo) Extraction and Identification

HUCMSCs were incubated with a FBS free culture medium for 72 h and centrifuged at 1,200 × g at 4°C for 25 min in order to remove the debris and dead cells, after which it was filtered using a 0.2-mm filter. Next, the cells were treated with ultra-centrifugation at 120,000 × g at 4°C for 2.5 h, followed by an additional round of ultra-centrifugation at 120,000 for 2 h and resuspended with PBS. Western blot analysis was performed in order to identify the characterization of the exosomes by measuring the expression of exosome specific markers HSP70 (ab79852), CD63 (ab216130), and CD9 (ab223052) as well as endoplasmic reticulum marker calnexin (ab10286) provided by Abcam Inc. (Cambridge, UK). Zetasizer Nano ZS (Malvern Instruments, Malvern, UK) was used to evaluate the particle size distribution of the exosomes. Transmission electron microscopy (TEM) was utilized to observe and analyze the morphology of the exosomes. The exosomes loaded onto carbon-coated nickel grids were negatively stained using 2% methylamine tungstate for 5 min. The staining was then examined under a JEM-1230 electron microscope (Nihon Denshi, Tokyo, Japan) at an accelerating voltage of 80 kV.

### Laser Scanning Confocal Microscope (LSCM)

Carboxyfluorescein diacetate succinimidyl ester (CFSE) dye (dilution ratio of 1:1,000) was uniformly mixed with 20 μg transfected HUCMSCs-exo suspension and permitted to stand at 37°C for 15 min. Next, the mixture was centrifuged at 100,000 × g for 70 min, and CFSE-labeled exosomes were co-cultured with the breast cancer cells, with the uptake of exosomes by the breast cancer cells observed under a LSCM at the 12th, 24th, and 48th h time intervals respectively.

### Co-culture of HUCMSCs-exo and Breast Cancer Cells

The exosomes were extracted from HUCMSCs transfected with NC-mimic, miR-148b-3p-mimic, NC-inhibitor, and miR-148b-3p-inhibitor, namely, Exo-NC-mimic, Exo-miR-148b-3p-mimic, Exo-NC-inhibitor, and Exo-miR-148b-3p-inhibitor, respectively. The extracted exosomes were co-cultured with breast cancer cells MDA-MB-231 for 48 h after the cell confluence in the 24-well plate reached 60%.

### Transwell Assay

Invasion assays were performed as follows: the Transwell plate (3,415, Corning Incorporated, Corning, NY, USA) was coated with 50 μL of diluted Matrigel gel (YB356234, Shanghai Yu Bo Biotech, Co, Ltd., Shanghai, China) and subsequently incubated for 2–3 h. The cells were then detached and prepared into a cell suspension using culture medium with 10% FBS at a density 10 × 10^5^ cells/mL. Next, 200 μL cell suspension was added into the apical chamber and 800 μL culture medium with 20% FBS was added into the basolateral chamber and cultured in a 37°C incubator for 20–24 h. The cells were then rinsed with formaldehyde for 10 min, stained with 0.1% crystal violet, and permitted to stand at room temperature for 30 min. Next, the cells on the surface were removed, followed by observation, photography, and counting under the guidance of an inverted microscope.

Additionally, the migration assay was conducted as follows: the cells were cultured for 16 h without Matrigel. Four power fields were randomly selected for cell counting.

### 5-Ethynyl-2'-deoxyuridine (EdU)

After 48-h transfection, the breast cancer cells MDA-MB-231 were incubated with EdU culture medium (A10044; Invitrogen^TM^, Thermo Fisher Scientific) for 2 h. Conventional steps were performed in accordance with the method from a previous study (17). The cells with a red-stained nucleus were regarded as positive cells. Three power fields were randomly selected under the guidance of a microscope to count the number of positive and negative cells. EdU labeling rate (%) = the number of positive cells/(the number of positive cells + negative cells) × 100%.

### Flow Cytometry

The breast cancer cells MDA-MB-231 were collected and subjected to the following experiments in strict accordance with the instructions of Annexin V-FITC/propidium iodide (PI) apoptosis detection kit (MA0220, Meilunbio, Dalian, China). Initially, the cells were counted. Next, 2–5 × 10^5^ cells/mL were centrifuged at 500 × g for 5 min. After the supernatant had been discarded, the cells were resuspended with 195 μL binding buffer working solution, incubated with 5 μL Annexin V-FITC for 10 min, and later 10 μL PI (20 μg/mL) for 5 min under conditions devoid of light. The blank control, PI simple staining and Annexin V-FITC single staining groups were established.

### Dual-Luciferase Reporter Gene Assay

TRIM59 sequence containing miR-148b-3p binding site and the mutant (MUT) sequence with the miR-148b-3p binding site mutated were constructed and inserted into the pGL3 Luciferase reporter vectors (E1751, Promega Corp., Madison, WI, USA), namely the PGL3-TRIM59 wild type (WT) and pGL3-TRIM59 MUT. The recombinant plasmids were co-transfected with miR-148b-3p mimic or NC plasmids into the HEK293T cells, respectively. After a 24-h period of transfection, the cells were lysed and centrifuged at 25,764 × g for 1 min. After the supernatant had been collected, the Dual-Luciferase® Reporter Assay System (E1910, Promega Corp., Madison, Wisconsin, USA) was used to determine the luciferase activity.

### RNA Isolation and Quantitation

The total RNA of the tissues or cells was extracted in accordance with the instructions of the TRIzol reagent kit (15596-018, Beijing Solarbio Life Sciences Co., Ltd., Beijing, China). The RNA concentration was subsequently determined. The primers were synthesized by Takara (Takara Holdings Inc., Kyoto, Japan) (Table 1). Reverse transcription was conducted based on the one-step method provided by the miRNA reverse transcription reagent kit (D1801, HaiGene, Harbin, China) and cDNA reverse transcription reagent kit (K1622, Beijing Yaanda Biological Technology Co., Ltd., Beijing, China). Real time quantitative polymerase chain reaction (qPCR) was performed using a fluorescent quantitation PCR instrument (ViiA 7, Daan Gene Co., Ltd., Guangzhou, China). U6 and β-actin were regarded as the endogenous controls. The fold changes were calculated based on relative quantification (the 2^−ΔΔ*Ct*^ method) (18).

**Table 1:** RT-qPCR primer sequences.

**Gene**	**Sequence (5^′^-3^′^)**
miR-148b-3p	F: CGGTCAGTGCATCACAGAA
	R: GTGCAGGGTCCGAGGT
TRIM59	F: CCCCCAAACCACGAGATCAA
	R: TGAGAGCATGGCAGTACACG
U6	F: CTCGCTTCGGCAGCACA
	R: AACGCTTCACGAATTTGCGT
β-actin	F: GGCACCACACCTTCTACAAT
	R: GTGGTGGTGAAGCTGTAGCC

*RT-qPCR, reverse transcription quantitative polymerase chain reaction; F, forward, R, reverse; TRIM59, tripartite motif59; miR-148b-3p, microRNA-148b-3p*.

### Western Blot Analysis

The total protein of the tissues or cells was extracted using radio-immunoprecipitation assay (RIPA) cell lysis buffer (R0010, Beijing Solarbio Life Sciences Co., Ltd., Beijing, China). The protein concentration of each sample was subsequently determined using a bicinchoninic acid (BCA) kit (20201ES76, Shanghai Yeason Biological Technology Co., Ltd., Shanghai, China). After separation by polyacrylamide gel electrophoresis, the protein was transferred onto the polyvinylidene fluoride membrane *via* the wet-transfer method and then sealed with 5% bovine serum albumin (BSA) for 1 h. Next, the membrane was incubated with the diluted primary antibodies mouse anti-human B-cell lymphoma-2 (Bcl-2) (ab182858, dilution ratio of 1:2,000), Bcl-xl (ab32370, dilution ratio of 1:1,000), Bcl2 Associated X protein (Bax) (ab32503, dilution ratio of 1:5,000), E-cadherin (ab15148, dilution ratio of 1:500), N-cadherin (ab18203, dilution ratio of 1:1,000), Vimentin (ab137321, dilution ratio of 1:1,000), TRIM59 (ab166793, dilution ratio of 1:800), and β-actin (ab8226, dilution ratio of 1:5,000) at 4°C overnight. All the aforementioned antibodies were purchased from Abcam Inc. (Cambridge, UK). The membranes were then rinsed three times with tris-buffered saline with Tween 20 (TBST) (5 min per wash), and reacted with the diluted Horse Reddish Peroxidase (HRP)-labeled goat anti-rabbit immunoglobulin G (IgG) (ab205718, dilution ratio of 1:20,000, Abcam Inc., Cambridge, UK) at room temperature for 1 h. The membranes were then subjected to an additional round of TBST washing and added with developing liquid for coloration. Finally, protein quantitative analyses were conducted using ImageJ 1.48u software (National Institutes of Health, Bethesda, Maryland, USA) based on the gray value ratio of each protein to β-actin.

### Immunohistochemistry

The paraffin-embedded tumor tissue sections from the nude mice were dewaxed and dehydrated with gradient ethanol. The sections were then repaired in antigen retrieval buffers and subsequently sealed with normal goat serum (C-0005, Shanghai Haoran Biological Technology Co., Ltd., Shanghai, China) at room temperature for 20 min. The sections were then added with primary mouse anti-human Ki-67 (ab833, dilution ratio of 1:50), TRIM59 (ab166793, dilution ratio of 1:150), E-cadherin (ab15148, dilution ratio of 1:30), N-cadherin (ab18203, dilution ratio of 1:300), and Vimentin (ab137321, dilution ratio of 1:200) overnight at 4°C. Afterwards, the sections were added with the secondary antibody goat anti-rabbit IgG (ab6785, dilution ratio of 1:1,000) at 37°C for 20 min. All the above-mentioned antibodies were procured from Abcam Inc. (Cambridge, UK). The sections were subsequently treated with HRP-labeled streptavidin (0343-10000U, Yi Mo Biological Technology Co., Ltd., Beijing, China) at 37°C for 20 min, followed by conventional DAB coloring and hematoxylin counter-staining. Under the guidance of a microscope, positive staining was scored based on a previously described method (19). Five high-power fields were randomly selected from each section, with the percentage of positively stained cells in each field of view was scored as follows: positive cells <10% are negative, positive cells ≧ 10 and <50% are positive, and the number of positive cells > 50% is strongly positive.

### Tumor Xenograft in Nude Mice

A total of 18 athymia nude mice (aged 4–6 weeks, Hunan SLAC Laboratory Animal Co., Ltd., Hunan, China) were randomly assigned into 3 groups (6 mice per group). Next, MDA-MB-231 cells (1 × 10^6^ cells/mouse) were injected into the mice through the mammary fat pad in order to establish breast cancer orthotopic transplantation tumor models. Next, 10^8^ exosomes in 100 μL of PBS were delivered into each nude mouse *via* tail intravenous injections on the 0th, 5th, 10th, 15th, and 20th days. Specifically, the nude mice were administered injections with Exo-NC-agomir and Exo-miR-148b-3p agomir or 100 μL PBS only. The nude mice were euthanized on the 28th day in order to collect and analyze the growth of tumors (volume and weight). The tumor volume was calculated based on the following formula: Volume = (Width^2^ × Length)/2. Total RNA and protein of tumor tissues were extracted in order to determine the expression of miR-148b-3p and TRIM59. Tumor tissues were routinely paraffin-embedded and the sections were subjected to immunohistochemistry.

### Statistical Analysis

All data were analyzed using the Statistic Package for Social Science (SPSS) 21.0 statistical software (IBM Corp. Armonk, NY, USA). Measurement data were expressed as mean ± standard deviation. The experiments were conducted independently in triplicates. The data among tumor tissues and adjacent normal tissues were analyzed using a paired *t* test, while data between two groups were analyzed using an unpaired *t* test. Comparisons among multiple groups were performed using one-way analysis of variance (ANOVA) with Tukey's *post hoc* test. Comparisons at different time points were conducted using repeated-measures ANOVA. A value of *p* < 0.05 was considered to be reflective of statistical significance.

## Results

### Poorly Expressed miR-148b-3p in Breast Cancer Tissues

Increasing evidence has proven that poor expression of miR-148b-3p is correlated with poor prognoses in breast cancer (20, 21). In order to determine the expression of miR-148b-3p in breast cancer, we collected breast cancer and adjacent normal tissues from 40 breast cancer patients whose information is shown in the Supplementary Table 1. Next, RT-qPCR was conducted to determine the expression of miR-148b-3p in breast cancer and adjacent normal tissues, and the results illustrated that the breast cancer tissues had a lower expression of miR-148b-3p compared to adjacent normal tissues (*p* < 0.05; Figure 1A). We subsequently uncovered that the expression of miR-148b-3p was reduced in breast cancer cell lines MDA-MB-231, MDA-MB-468, MCF-7, and MDA-MB-453 when compared to the normal breast epithelial cell line MCF-10A, with the lowest expression in MDA-MB-231 (*p* < 0.05; Figure 1B). Hence, the MDA-MB-231 cell line was selected for subsequent experimentation. The results demonstrated that miR-148b-3p was poorly expressed in breast cancer.

**Figure 1:** Reduced miR-148b-3p expression was detected in breast cancer. **(A)** The expression of miR-148b-3p in breast cancer and adjacent normal tissues was determined by RT-qPCR (ANT: adjacent normal tissues = 40; BC: breast cancer tissues = 40); *p < 0.05. **(B)** The expression of miR-148b-3p in normal breast epithelial cell line MCF-10A, breast cancer cell lines MDA-MB-231, MDA-MB-468, MCF-7, and MDA-MB-453 was determined by RT-qPCR; *p < 0.05, compared with MCF-10A. The data were expressed as mean ± standard deviation; data comparisons between breast cancer and adjacent normal tissues were analyzed using paired *t* test; comparisons among multiple groups were analyzed by one-way ANOVA (Tukey's *post hoc* test); *n* = 3. miR-148b-3p, microRNA-148b-3p; RT-qPCR, reverse transcription quantitative polymerase chain reaction; ANOVA, analysis of variance.

### miR-148b-3p Inhibited Cell Proliferation, Invasion and Migration, While Promoting Cell Apoptosis in Breast Cancer

In order to examine the effects associated with miR-148b-3p on the biological characteristics of breast cancer cells *in vitro*, we transfected MDA-MB-231 cells with miR-148b-3p mimic or miR-148b-3p inhibitor to conduct functional experiments. The results revealed an elevated expression of miR-148b-3p in the cells transfected with miR-148b-3p mimic, when compared with cells transfected with NC-mimic and NC-inhibitor, while those transfected with miR-148b-3p inhibitor exhibited decreased miR-148b-3p expression (*p* < 0.05; Figure 2A).

**Figure 2:** miR-148b-3p served as an inhibitor of cell proliferation, invasion and migration and a promoter of apoptosis in MDA-MB-231 cells. **(A)** The expression of miR-148b-3p in MDA-MB-231 cells following transfection with NC-mimic, miR-148b-3p mimic, NC-inhibitor and miR-148b-3p inhibitor were measured by RT-qPCR; **(B-E)**, proliferation **(B)**, invasion **(C)**, migration **(D)**, and apoptosis **(E)** of MDA-MB-231 cells following transfection with NC-mimic, miR-148b-3p mimic, NC-inhibitor and miR-148b-3p inhibitor were detected by EdU assay (× 200), Transwell assay (× 400) and flow cytometry, respectively. **(F)** Protein levels of E-cadherin, N-cadherin, Vimentin, Bcl-2, Bax, and Bcl-xl in MDA-MB-231 cells following transfection with NC-mimic, miR-148b-3p mimic, NC-inhibitor and miR-148b-3p inhibitor were determined by Western blot analysis. The data were expressed as mean ± standard deviation; pairwise comparisons between two groups were analyzed using unpaired *t* test; *p < 0.05; *n* = 3. miR-148b-3p, microRNA-148b-3p; NC, negative control, RT-qPCR, reverse transcription quantitative polymerase chain reaction; Bcl-2, B cell leukemia/lymphoma 2; Bax, Bcl2 associated X protein.

Next, cell vitality, invasion, and migration abilities, as well as the rate of apoptosis following transfection, were evaluated by EdU, Transwell assay and flow cytometry, respectively. The results revealed that transfection with miR-148b-3p mimic triggered a decline in MDA-MB-231 cell viability, invasion and migration abilities as well as increased apoptosis, which was contradictory to the changes elicited by inhibition of miR-148b-3p (*p* < 0.05; Figures 2B–E).

Next, Western blot analysis was conducted to determine the protein expression of epithelial-mesenchymal transition (EMT)-related proteins (E-cadherin, N-cadherin and Vimentin) and apoptosis-related proteins (Bcl-2, Bax, and Bcl-xl) in the MDA-MB-231 cells following transfection. The results obtained revealed up-regulated protein levels of E-cadherin and Bax, as well as down-regulated protein levels of N-cadherin, Vimentin, Bcl-2, and Bcl-xl in the cells transfected with miR-148b-3p mimic, while an opposite trend was identified in those transfected with miR-148b-3p inhibitor (*p* < 0.05; Figure 2F).

Taken together, the findings confirmed that miR-148b-3p inhibited cell proliferation, invasion, and migration but enhanced cell apoptosis in breast cancer.

### miR-148b-3p Negatively Regulated TRIM59 in Breast Cancer

Bioinformatics software (miRanda, TargetScan, and miRbase) was applied to predict the potential target genes of miR-148b-3p, which revealed TRIM59 as a potential target gene of miR-148b. Online analysis in TargetScan website confirmed the presence of a special binding area between the gene sequence of TRIM59 and miR-148b-3p (Figure 3A). Next a dual luciferase reporter gene assay was performed to verify this relationship. The results revealed that cells co-transfected with TRIM59-WT and miR-148b-3p mimic exhibited reduced luciferase activity (*p* < 0.05), while no significant differences were detected in the luciferase activity of TRIM59-MUT (*p* > 0.05). These findings suggested that miR-148b-3p could specifically bind to TRIM59 gene (Figure 3B).

**Figure 3:** TRIM59 was verified as the target gene of miR-148b-3p. **(A)** The binding site of miR-148b-3p and TRIM59 was predicted by the online website TargetScan. **(B)** The luciferase activity of TRIM59-WT and TRIM59-MUT following transfection with NC-mimic and miR-148b-3p mimic was detected by dual luciferase reporter gene assay. **(C,D)** The mRNA and protein expression of TRIM59 in MDA-MB-231 cells following transfection with NC-mimic, miR-148b-3p mimic, NC-inhibitor and miR-148b-3p inhibitor was measured by RT-qPCR and Western blot analysis, respectively. **(E)** The mRNA expression of TRIM59 in breast cancer and adjacent normal tissues was measured by RT-qPCR (ANT: adjacent normal tissues = 40; BC: Breast cancer tissues = 40). **(F)** The correlation analysis of TRIM59 and miR-148b-3p expression. **(G)** TRIM59 expression in breast cancer and adjacent normal tissues detected by immunohistochemical staining (× 400). **(H,I)** The mRNA and protein expression patterns of TRIM59 in MDA-MB-231 and MCF-10A cells was measured by RT-qPCR and Western blot analysis, respectively. The data were expressed as mean ± standard deviation; data comparisons between breast cancer and adjacent normal tissues were analyzed using paired *t* test; comparisons between two groups were analyzed by unpaired *t* test; *p < 0.05; *n* = 3. miR-148b-3p, microRNA-148b-3p; RT-qPCR, reverse transcription quantitative polymerase chain reaction; NC, negative control, TRIM59, tripartite motif59.

Next, the targeting relationship between miR-148b-3p and TRIM59 was further verified by perturbing the expression of miR-148b-3p in MDA-MB-231. It was found that the mRNA and protein expression of TRIM59 was notably decreased following miR-148b-3p mimic transfection, while an increase was identified by RT-qPCR and Western blot analyses following miR-148b-3p inhibitor transfection (*p* < 0.05; Figures 3C,D). These results provided verification that the expression of TRIM59 was negatively regulated by miR-148b-3p.

RT-qPCR and immunohistochemistry were employed to determine the expression of TRIM59 in the breast cancer and adjacent normal tissues. The results revealed that the breast cancer tissues exhibited a higher expression of TRIM59, when compared to the adjacent normal tissues (*p* < 0.05; Figures 3E,G). Furthermore, a correlation analysis revealed that the expression of TRIM59 was negatively correlated with the expression of miR-148b-3p (Figure 3F). Next, RT-qPCR and Western blot analysis were conducted again in order to determine the expression of TRIM59 in breast cancer cell line MDA-MB-231 and normal breast epithelial cell line MCF-10A. The results illustrated that the MDA-MB-231 cell line presented with up-regulated expression of TRIM59 compared to the MCF-10A cell line (*p* < 0.05; Figures 3H,I). In conclusion, these findings confirmed that TRIM59 was the target gene of miR-148b-3p and was further highly expressed in breast cancer.

### miR-148b-3p Modulated TRIM59 to Suppress Cell Proliferation, Invasion and Migration, and Enhance Cell Apoptosis in Breast Cancer

Recent studies have indicated that high expression of TRIM59 in breast cancer is associated with poor prognoses (16, 22, 23). In order to verify whether miR-148b-3p could exert its effects through inhibiting TRIM59, experiments with gain- or loss-of-function of TRIM59 in MDA-MB-231 cells were conducted, and miR-148b-3p mimic was employed to perturb the expression of TRIM59. EdU, Transwell assay, and flow cytometry results demonstrated that the overexpression of TRIM59 brought about a marked increase in viability, invasion and migration, but reduced apoptosis of MDA-MB-231 cells. In addition, inhibition of TRIM59 resulted in contrasting regulatory effects; however, the overexpression of miR-148b-3p reversed the pro-proliferation, pro-invasion, pro-migration, and anti-apoptotic effects of TRIM59 (*p* < 0.05; Figures 4A–D). Furthermore, Western blot analysis revealed that the up-regulation of TRIM59 expression elevated the protein levels of N-cadherin, Vimentin, Bcl-2, and Bcl-xl while it inhibited those of E-cadherin and Bax in MDA-MB-231 cells, but TRIM59 inhibition led to opposite results. Notably, the regulatory effects of TRIM59 on the aforementioned proteins were found to be reversed by enhancement of miR-148b-3p (*p* < 0.05; Figure 4E). Taken together, miR-148b-3p can down-regulate TRIM59, thereby inhibiting cell proliferation, invasion, and migration while promoting apoptosis in breast cancer.

**Figure 4:** miR-148b-3p played an inhibitory role in cell proliferation, invasion and migration and a stimulatory role in apoptosis of breast cancer cells. **(A–D)**, proliferation **(A)**, invasion **(B)** and migration **(C)**, and apoptosis **(D)** of MDA-MB-231 cells following transfection with TRIM59-NC, TRIM59, siRNA-NC, siRNA-TRIM59, or co-transfection with miR-148b-3p mimic and TRIM59-NC, miR-148b-3p mimic and TRIM59 were evaluated by EdU assay (× 200), Transwell assay (× 400) and flow cytometry, respectively. **(E)** Protein levels of E-cadherin, N-cadherin, Vimentin, Bcl-2, Bax and Bcl-xl in MDA-MB-231 cells following transfection with TRIM59-NC, TRIM59, siRNA-NC, siRNA-TRIM59, or co-transfection with miR-148b-3p mimic and TRIM59-NC, miR-148b-3p mimic and TRIM59 were determined by Western blot analysis. The data were expressed as mean ± standard deviation; comparisons between two groups were analyzed by using unpaired *t* test; *p < 0.05; *n* = 3; miR-148b-3p, microRNA-148b-3p; NC, negative control, TRIM59, tripartite motif59.

### Identification and Isolation of HUCMSCs and HUCMSCs-exo

Flow cytometry was employed to detect the expression patterns of surface markers of HUCMSCs. The results showed that the cells expressed typical CD marker profiles of the following HUCMSCs: positive for CD29 (100.0%), CD44 (100.0%), CD73 (99.3%), CD90 (99.7%), and HLA-A,B,C (100.0%); while negative for CD14 (3.4%), CD19 (16.3%), CD34 (19.6%), CD45 (19.2%), and HLA-DR (17.1%) (Figure 5A). The results obtained confirmed that the isolated cells from human umbilical cord were HUCMSCs.

**Figure 5:** Identification of HUCMSCs and HUCMSCs-exo. **(A)** The expression of surface markers of HUCMSCs (CD29, CD44, CD73, CD90, HLA-A,B,C, CD14, CD19, CD34, CD45, and HLA-DR) was detected by flow cytometry. **(B)** The morphology of HUCMSCs-exo was observed under TEM (scale bar = 200 nm). **(C)** Particle size distribution of HUCMSCs-exo was analyzed by Zetasizer Nano ZS. **(D)** The expression of HUCMSCs-exo surface markers (HSP70, CD63, and CD9) was determined by Western blot analysis. The data were expressed as mean ± standard deviation; comparisons between two groups were analyzed by using unpaired *t* test; *n* = 3; HUCMSCs, human umbilical cord mesenchymal stem cells; miR-148b-3p, microRNA-148b-3p; TEM, transmission electron microscopy; NC, negative control, TRIM59, tripartite motif59.

Next, characterization of the exosomes from HUCMSCs was identified. TEM imaging identified a gathering of round or oval-shaped membrane vesicles with notable heterogeneity in size and a diameter of 40–150 nm, where membranous structure was detected in the peripheral area and component of low electronic density was detected in the central part (Figure 5B). Furthermore, Zetasizer Nano ZS particle size analysis revealed that the diameter of the HUCMSCs-exo was ~61.58 nm (Figure 5C). Western blot analysis was performed to detect the expression of exosome surface markers (HSP70, CD63, and CD9), which revealed a higher expression of HSP70, CD63, and CD9 in HUCMSCs-exo than in HUCMSCs (Figure 5D). Taken together, these results indicated that the HUCMSCs-exo were successfully extracted.

### HUCMSCS-exo-Carrying miR-148b-3p Inhibited Cell Proliferation, Invasion, and Migration While Promoted Cell Apoptosis in Breast Cancer

In order to verify whether breast cancer cell line MDA-MB-231 could uptake HUCMSCs-exo, CFSE-labeled HUCMSCs-exo were co-cultured with MDA-MB-231 and photographed under LSCM at 12th, 24th, and 48th h time intervals, respectively. With the extension of co-culture time, a progressive increase in cells exhibiting green fluorescence was identified, highlighting an increase in the number of HUCMSCs-exo internalized by MDA-MB-231 cells, with a more noticeable increase at the 48th h time interval (Figure 6A).

**Figure 6:** HUCMSCs-exo-transporting miR-148b-3p suppressed cell proliferation, invasion and migration, but accelerated cell apoptosis. Exosomes were extracted from HUCMSCs transfected with NC-mimic, miR-148b-3p-mimic NC-inhibitor and miR-148b-3p-inhibitor, namely, Exo-NC-mimic, Exo-miR-148b-3p-mimic, Exo-NC-inhibitor, and Exo-miR-148b-3p-inhibitor, respectively. MDA-MB-231 cells were co-cultured with HUCMSCs-exo or not (control). **(A)** Uptake of HUCMSCs-exo by MDA-MB-231 cells at various time intervals (12th, 24th, and 48th h); green represented CFSE-labeled exosomes and blue represented DAPI-labeled nucleus (× 400). **(B)** The expression of miR-148b-3p and TRIM59 in MDA-MB-231 cells was determined by RT-qPCR; C-E, MDA-MB-231 cell proliferation **(C)**, invasion and migration **(D)**, and apoptosis rate **(E)** were assessed by EdU assay (× 200), Transwell assay (× 400) and flow cytometry. **(F)** Protein levels of E-cadherin, N-cadherin, Vimentin, Bcl-2, Bcl-xl, and Bax in MDA-MB-231 cells was determined by Western blot analysis. The above data was expressed as mean ± standard deviation; comparisons between two groups were analyzed using unpaired *t* test; *p < 0.05; *n* = 3. HUCMSCs, human umbilical cord mesenchymal stem cells; HUCMSCs-exo, HUCMSCs-derived exosomes; miR-148b-3p, microRNA-148b-3p; RT-qPCR, reverse transcription quantitative polymerase chain reaction; NC, negative control.; EdU, 5-ethynyl-2'-deoxyuridine; Bcl-2, B cell leukemia/lymphoma 2; Bax, Bcl2 associated X protein; TRIM59, tripartite motif59.

Next, exosomes were extracted from HUCMSCs transfected with miR-148b-3p mimic or inhibitor to verify whether miR-148b-3p could exert its inhibitory effect on breast cancer by HUCMSCs-exo. HUCMSCs-exo were co-cultured with MDA-MB-231 cells. RT-qPCR revealed that MDA-MB-231 cells co-cultured with HUCMSCs-exo derived from the HUCMSCs transfected with miR-148b-3p mimic presented with increased miR-148b-3p and decreased TRIM59 expression, while reduced miR-148b-3p and increased TRIM59 expression were detected in the MDA-MB-231 cells co-cultured with HUCMSCs-exo derived from the HUCMSCs transfected with miR-148b-3p inhibitor (*p* < 0.05; Figure 6B). The aforementioned results demonstrated that HUCMSCs-exo could effectively deliver miR-148b-3p to breast cancer cells.

The results obtained from EdU, Transwell assay and flow cytometry revealed that HUCMSCs-exo carrying miR-148b-3p induced reductions in viability, invasion, and migration, and an increase in the apoptotic ability of MDA-MB-231 cells, while the inhibition of HUCMSCs-derived exosomal miR-148b-3p exerted a contrasting effects (*p* < 0.05; Figures 6C–E). Furthermore, Western blot analysis demonstrated that HUCMSCs-exo carrying miR-148b-3p initiated elevations in the protein levels of E-cadherin and Bax, and reductions in the protein levels of TRIM59, N-cadherin, Vimentin, Bcl-2, and Bcl-xl, all of which were opposite to that induced by inhibition of HUCMSCs-derived exosomal miR-148b-3p (*p* < 0.05; Figure 6F). Hence, we concluded that HUCMSCs-exo-carrying miR-148b-3p could inhibit cell proliferation, invasion, and migration, while increasing the apoptosis of breast cancer cells.

### HUCMSCs-exo-Carrying miR-148b-3p Inhibited Tumor Formation and EMT in Nude Mice

In order to further verify the inhibitory effect associated with HUCMSCs-exo-carrying miR-148b-3p on tumor formation in xenograft tumors of nude mice *in vivo*, MDA-MB-321 cells were injected into nude mice *via* the mammary fat pad to establish primary xenograft tumor models, and exosomes secreted from HUCMSCs were intravenously injected into nude mice *via* the tail vein. It was shown that the delivery of Exo-NC-agomir and Exo-miR-148b-3p agomir brought about a notable decrease in tumor volume and weight in the nude mice (*p* < 0.05; Figures 7A,B). RT-qPCR indicated increased miR-148b-3p expression and reduced TRIM59 expression following the delivery of Exo-miR-148b-3p agomir (*p* < 0.05; Figure 7C).

**Figure 7:** Exosomal miR-148b-3p suppressed tumor formation and EMT in nude mice. After establishment of primary xenograft tumor models by mammary fat pad injection of MDA-MB-321 cells, tumor bearing nude mice were subjected to injection of PBS (control), Exo-NC-agomir or Exo-miR-148b-3p agomir. **(A,B)** Observation and records of tumor volume and weight in nude mice. **(C)** The expression of miR-148b-3p and TRIM59 in tumor tissues was determined by RT-qPCR. **(D)** Protein levels of TRIM59, E-cadherin, N-cadherin, Vimentin, Bcl-2, Bcl-xl, and Bax were measured by Western blot analysis. **(E)** Levels of TRIM59, Ki-67, E-cadherin, N-cadherin, and Vimentin were detected by immunohistochemistry (× 400). The above data was expressed as mean ± standard deviation; comparisons between two groups were analyzed using unpaired *t* test; comparisons among multiple groups are analyzed by repeated measures ANOVA; *p < 0.05; *n* = 6 for animal grouping; *n* = 3. miR-148b-3p, microRNA-148b-3p; RT-qPCR, reverse transcription quantitative polymerase chain reaction; NC, negative control; Bcl-2, B cell leukemia/lymphoma 2; Bax, Bcl2 associated X protein; TRIM59, tripartite motif59; ANOVA, analysis of variance.

Additionally, Western blot analysis showed that the delivery of Exo-miR-148b-3p agomir caused an elevation in the protein levels of E-cadherin and Bax, while reducing those of TRIM59, N-cadherin, Vimentin, Bcl-2, and Bcl-xl (*p* < 0.05; Figure 7D).

Finally, immunohistochemistry revealed that the level of E-cadherin was elevated, while the levels of Ki-67, TRIM59, N-cadherin, and Vimentin were diminished after the delivery of Exo-miR-148b-3p agomir (*p* < 0.05; Figure 7E). In conclusion, xenograft tumor growth and EMT in nude mice were inhibited by HUCMSCs-exo-carrying miR-148b-3p.

## Discussion

Despite significant advancements made in cancer therapeutic and diagnostic approaches, breast cancer remains one of the most prevalent malignant tumors affecting millions of women worldwide (1). miRs have been strikingly highlighted as diagnostic, prognostic, and therapeutic targets for breast cancer (24, 25). Recent studies have indicated that exosomes are derived from various types of cells and contain parent cells-secreted miRs, lipids, and proteins (26, 27). The current study aimed to elucidate the role by which HUCMSC-exo carrying miR-148b-3p influences breast cancer. Collectively, our findings provided evidence demonstrating that HUCMSC-exo carrying miR-148b-3p could function as a suppressor of breast cancer by down-regulating the expression of TRIM59.

A notable finding of the current study revealed that miR-148b-3p was poorly expressed in breast cancer and functioned as an anti-tumor miR by suppressing cancer cell growth, migrating, and invasive capabilities of cancer cells, in addition to promoting cancer cell apoptosis. Mangolini et al. concluded that patients with breast cancer exhibited decreased expression of miR-148b-3p, consistent with that of the current study (20). Similarly, the down-regulation of miR-148b-3p expression has been previously linked with unsatisfactory survival outcomes in patients with breast cancer (21). Furthermore, the overexpression of miR-148b-3p has been previously suggested to be implicated in the inhibition of cell proliferation and invasion, and promotion of cell apoptosis in human pituitary adenomas, while we uncovered a similar effect on breast cancer cells in the current study (28). Additionally, the overexpression of miR-148a is widely considered to play a contributory role in suppressing the invasion and migration of breast cancer cell lines MCF-7 and MDA-MB-231 (29). Moreover, the current study revealed that TRIM59 gene was highly expressed in breast cancer. TRIM59 gene has been previously suggested as a novel multiple tumor marker for tumorigenesis detection during the initial stages, highlighting its potential as a therapeutic target for cancer diagnosis and therapy (16). Furthermore, a recent study also noted the up-regulated expression of TRIM59 in breast cancer cells, which was consistent with our findings (22). Meanwhile, another study has revealed that TRIM59 down-regulation contributes to inhibition of proliferation, migration, and invasion in breast cancer, all of which are crucial factors in the treatment of breast cancer (23). Consistently, TRIM59 expression knock-down facilitates tumor cell apoptosis and prevents tumorigenesis (30). Moreover, the current study revealed that miR-148b-3p targets TRIM59 and negatively regulates its expression. Hence, these evidences indicate that miR-148b-3p overexpression inhibits cell proliferation, invasion, and migration, while promoting cell apoptosis in breast cancer by down-regulating TRIM59.

Furthermore, our findings provided evidence indicating that miR-148b-3p, which can be subsequently transferred into breast cancer cells *via* exosomes derived from HUCMSCs, exerts its function by targeting TRIM59. Exosomes are membrane vesicles that can be derived from stromal and tumor cells and play a role in tumorigenesis, contributing to development of exosomes-based therapies (31, 32). Meanwhile, various cell types-derived exosomal tumor-suppressive miRs have also been documented to exert inhibitory effects on tumor growth (33). For instance, miR-100 has been shown to act as a tumor suppressor by restraining breast cancer cell migration and invasion (34). Likewise, MSCs-derived exosomes overexpressing miR-100 contribute to the suppression of angiogenesis in breast cancer (35). Moreover, the beneficial effects of miR-148b have been documented to inhibit tumor cell metastasis and restrain tumor growth in breast cancer (36). Furthermore, a previous study revealed that the inhibition of breast cancer cell proliferation, migration, and invasion could be triggered by TRIM59 knockdown (23). Those mentioned above are partially consistent with the most crucial finding of the current study, whereby HUCMSC-derived exosomes carrying miR-148b-3p were identified to inhibit cell proliferation, invasion, and migration, while promoting cell apoptosis in breast cancer by down-regulating TRIM59.

Taken together, HUCMSC-exo carrying miR-148b-3p have the potential to serve as a promising miR-targeted therapy for breast cancer patients, due to its inhibitory effects on tumor cell proliferation, invasion, and migration, as well as its stimulatory effect on cell apoptosis in breast cancer (Figure 8). Our investigation of HUCMSC-exo carrying miR-148b-3p yielded promising results and an enhanced understanding regarding its potential as a breast cancer therapeutic strategy. However, the research is still at the preclinical stage. In addition, the underlying role and mechanism of miR-148b-3p in breast cancer stills remain to be elucidated. Thus, further investigations are needed to explore the relevant intrinsic mechanisms.

**Figure 8:** miR-148b-3p was delivered into breast cancer cells through HUCMSCs-exo. miR-148b-3p inhibited cell proliferation and EMT while promoted cell apoptosis by suppressing TRIM59 in breast cancer cells. HUCMSCs, human umbilical cord mesenchymal stem cells; HUCMSCs-exo, HUCMSCs-derived exosomes; miR-148b-3p, microRNA-148b-3p; Bcl-2, B cell leukemia/lymphoma 2; Bax, Bcl2 associated X protein; EMT, epithelial-mesenchymal transition.

## Data Availability Statement

The raw data supporting the conclusions of this manuscript will be made available by the authors, without undue reservation, to any qualified researcher.

## Ethics Statement

The current study was performed in strict accordance with the recommendations in the Guide for the Care and Use of Laboratory Animals of the National Institutes of Health. All experiment protocols were conducted with the approval of the Ethics Committee of the First Affiliated Hospital of Zhengzhou University. All participants signed informed consent prior to the study. All study protocols were performed in strict adherence to the ethical principles for medical research involving human subjects of the Helsinki Declaration.

## Author Contributions

LY, YL, YQ, LL, and HL: conception and design of the study and approval of the manuscript. LY, YL, and YQ: performed the experiments. LY and HL: data analysis. YL, YQ, and LL: drafted the paper.

### Conflict of Interest

The authors declare that the research was conducted in the absence of any commercial or financial relationships that could be construed as a potential conflict of interest.
